The article "MCFN: A Multichannel Fusion Network for Sleep Apnea Syndrome Detection" was published in 2023. Journal: J Healthc Eng.

# MCFN: A Multichannel Fusion Network for Sleep Apnea Syndrome Detection

**DOI:** 10.1155/2023/5287043

**Published:** 2023-01-23

**Authors:** Xingfeng Lv, Jinbao Li, Qianqian Ren

**Affiliations:** ^1^College of Electronic Engineering, Heilongjiang University, Harbin 150080, China; ^2^Department of Computer Science and Technology, Heilongjiang University, Harbin 150080, China; ^3^Shandong Artificial Intelligence Institute, Qilu University of Technology (Shandong Academy of Science), Jinan 250353, China

## Abstract

Sleep apnea syndrome (SAS) is the most common sleep disorder which affects human life and health. Many researchers use deep learning methods to automatically learn the features of physiological signals. However, these methods ignore the different effects of multichannel features from various physiological signals. To solve this problem, we propose a multichannel fusion network (MCFN), which learns the multilevel features through a convolution neural network on different respiratory signals and then reconstructs the relationship between feature channels with an attention mechanism. MCFN effectively fuses the multichannel features to improve the SAS detection performance. We conducted experiments on the Multi-Ethnic Study of Atherosclerosis (MESA) dataset, consisting of 2056 subjects. The experiment results show that our proposed network achieves an overall accuracy of 87.3%, which is better than other SAS detection methods and can better assist sleep experts in diagnosing sleep disorders.

## 1. Introduction

Sleep apnea syndrome (SAS) is a common sleep-breathing disorder characterized by repetitive events of complete or partial cessation of breathing during sleep [1]. SAS often occurs in men and women aged 30 to 60 years or older [2]. The main symptoms of SAS are daytime sleepiness, tiredness, inattention, and so on. Most SAS patients are undiagnosed and untreated which may lead to health problems such as heart and brain diseases [3–6].

SAS includes two important sleep events: obstructive sleep apnea (OSA) and hypopnea. According to an American Academy of Sleep Medicine (AASM) manual [7], OSA is scored when there is a 90% or more reduction in the prevent baseline of the airflow amplitude. However, there is a continued respiratory effort in the thoracic and abdominal belts. Hypopnea is scored when there is a 30% or more reduction in the preevent baseline of the airflow and 3% or more significant oxygen desaturation from the preevent baseline. Every OSA and hypopnea event lasts longer than 10 s. Normal sleep is scored when there is no OSA and hypopnea event or their duration time is less than 10 s.

Diagnosing SAS traditionally uses polysomnography (PSG), which is the gold standard. PSG can measure several signals, such as respiratory, electrocardiography (ECG), blood oxygen saturation, electroencephalography (EEG), and body movement signals. However, it is expensive and inconvenient because the patients need to attach a variety of sensors to their bodies. Moreover, it is time-consuming due to the manual analysis of signals. Therefore, it is necessary to propose alternative methods to automatic SAS detection using fewer physiological signals.

Various physiological signals have been used to detect sleep events [8–10]. Among these signals, respiratory signals can directly reflect the breathing situation during sleep [11]. The respiratory signal can be measured directly from the airflow sensor and thoracic and abdominal belts. Some methods have been used for SAS detection, such as threshold, support vector machine (SVM), logical regression (LR), and *k* nearest-neighbor (*k*-NN) [12–16]. These methods extracted the time domain, frequency domain, and other nonlinear features from physiological signals. However, manual feature extraction is difficult to perform in noisy signals and requires domain knowledge.

Deep learning networks are alternatives as they can learn informative features without prior domain knowledge. Many researchers use long- and short-term memory (LSTM) and convolutional neural networks (CNNs) to classify physiological signals [17–32]. In particular, CNN is a popular class of deep learning networks that can automatically learn and find features from physiological signals. Haidar et al. [22] have demonstrated the efficacy of CNN models in classifying apnea or hypopnea events using airflow respiratory signals, with an accuracy of 77.6%. When a wavelet spectrogram of airflow respiratory signals input the network, the accuracy was 79.8%. If we use abdominal and thoracic respiratory signals simultaneously, the performance can reach 83.5% [23]. Urtnasan et al. [24] proposed a method for automated OSA detection from a single-lead ECG using CNN. Choi et al. [25] used CNN and a single-channel nasal pressure signal to detect the real-time apnea-hypopnea event. Nasal pressure signals were adaptively normalized and segmented by sliding a 10 s window at 1 s intervals. Many researchers use the LSTM model for SAS detection to learn the temporal features of sleep events. Van Steenkiste et al. [26] used LSTM to detect sleep apnea from raw respiratory signals, obtaining 77.2% accuracy. Elmoaqet et al. [27] used LSTM and bidirectional long-short-term memory (Bi-LSTM) to detect three sleep events and got an average accuracy of 83.6%. Yu et al. [32] proposed a method of sleep staging based on EEG signals combined with sleep apnea-hypopnea syndrome classification, which significantly reduced the rate of false positives that appear in the waking period. The data preprocessed by the sliding window were manipulated by LSTM and CNN to identify distinct various sleep events. Although these networks can automatically extract and learn deep-level features from physiological signals, there are still some shortcomings. First, they only focus on extracting deep features, ignoring the effect of shallow features, which can provide rich information for sleep events. Our initial conference paper solved this problem using a multilevel feature fusion network in [33]. Second, these networks did not consider the impact of channel features obtained by different respiratory signals. Some channel features can clearly distinguish sleep events, while others have little effect on SAS detection. We propose a multichannel fusion network (MCFN) to address this problem. MCFN effectively utilizes the shallow features of respiratory signals and fuses the multichannel features by an attention mechanism. We design a multichannel fusion block to calibrate the feature channel of various respiratory signals adaptively. Since the significance of each respiratory signal feature channel is different, this block can automatically obtain the importance of each feature channel, selectively enhance the useful channel feature, and restrain the useless ones. We evaluate our proposed network on a publicly available dataset with 2056 subjects. The MCFN can achieve an overall accuracy of 87.3%.

## 2. Material and Methods

MCFN can effectively fuse the features of different levels and channels. This network mainly includes signal preprocessing, multilevel feature concatenation, and multichannel attention fusion. We show the framework in Figure 1. First, we segment the various respiratory signals into a series of the 30 s length of epochs. The preprocessing block standardizes the respiratory signals, and each epoch is labeled as an event of OSA, hypopnea, and normal sleep according to the AASM guidelines. Second, the multilevel feature concatenation block obtains abundant features from shallow and deep layers through skip connections. Shallow features also contain some valuable identification information. Third, the multichannel fusion block uses an attention mechanism to learn different weights. The channel features that significantly affect SAS detection can obtain larger weights; otherwise, they get smaller weights. Finally, the feature vectors are input into two convolution layers and the max-pooling layer. The sleep classification is performed in the fully connected layer by sigmoid activation functions. In the following subsections, we detail the main block of this network.

### 2.1. Dataset

We conducted our experiments on a large dataset called the Multi-Ethnic Study of Atherosclerosis (MESA) [28, 29]. This dataset is retrieved from the National Sleep Research Resource (NSRR). NSRR is a new National Heart, Lung, and Blood Institute resource designed to provide extensive data resources to the sleep research community. MESA contains PSG recordings of 2056 subjects. The subjects, aged 45 to 84, come from different ethnic groups, including black, white, Hispanic, and Chinese men and women. Each PSG recording included various physiological signals such as EEG, respiration signals, and ECG. Our network only used three types of respiratory signals extracted from nasal thermal sensors and conductive belts around the thorax and abdomen. The sampling frequency of these signals is 32 Hz. Sleep experts labeled the start time and duration time of OSA and hypopnea events.

### 2.2. Data Preprocessing

In our network, three types of respiratory signals need to be preprocessed. First, we delete some subjects from the dataset which only contain normal sleep events. Second, due to different detection environments and equipment, the amplitude of each respiratory signal is very different. Therefore, the respiratory signal is individually standardized by subtracting the mean and dividing it by the standard deviation. Finally, according to the time of each sleep event, each 30 s epoch was labeled as OSA, hypopnea, or normal sleep event. If the epoch contains only obstructive sleep apnea or hypopnea lasting more than 10 seconds, it is labeled OSA or hypopnea. We excluded the epoch with obstructive sleep apnea and hypopnea events lasting more than 10 seconds. If an epoch contains obstructive sleep apnea or hypopnea events lasting less than 10 seconds, it is labeled as normal sleep.

We also need to consider the balance classification of sleep events in preprocessing blocks. Typically, sleep events such as normal sleep are more than OSA or hypopnea. When learning a detection network with imbalanced classes, the result detects the most frequent sleep events. One way to address this issue is to employ balanced sampling. We randomly select the same number from the majority sleep event as the minority sleep event and then feed the network with batches of data that contain as many epochs from each sleep event.

### 2.3. Multilevel Feature Concatenation Block

A simple CNN architecture has been used for SAS detection [23, 33]. It was composed of convolution, pooling, and classification layers. The convolution layer extracts a feature map by applying a filter to the input respiratory signal. The pooling layer makes the feature more distinct and reduces the amount of data. The convolution layer can filter out some high-frequency information and make the signal smoother. In Figure 2, the partial feature map of the airflow respiratory signal after four convolution layers is shown. We find that with the increase of convolution layers, the receptive field of features becomes larger, and more high-frequency information is filtered. Although some networks use deep-level features to detect SAS, some high-frequency features are lost. Multilevel feature concatenation is realized through five skip connections to keep more high-frequency features in the network.

The multilevel feature concatenation block includes four convolution layers, two pooling layers, five skip connections, and one concatenation. We detail the parameters of different layers, which are summarized in Table 1. Each convolution layer has 32 filters with a rectified linear unit activation function, and each max-pooling layer has a pool size of (1, 2) with two strides. The convolutional kernel size is (1, 3) with three strides or (1, 2) with two strides. Following each convolution and pooling layer, the features of this level are obtained by average pooling to down-sampling. Then, these features are concatenated to generate multilevel feature maps. These features include shallow and deep features and provide more basic information. They can improve detection performance.

### 2.4. Multichannel Attention Fusion Block

Different respiratory signals such as airflow, thoracic, and abdominal have additional predictive power for SAS detection [27]. We fuse the multichannel features with an attention mechanism to fully use multilevel features from three types of respiratory signals. This block adaptively recalibrates channel-wise feature responses by explicitly modeling interdependencies between channels. It can learn to emphasize informative features and restrain less useful ones selectively.

As shown in Figure 1, we obtain the *C* × *W* × *H* features through the multilevel feature concatenation block, where *C* is the number of channels, and each channel contains *W* × *H* features. Each respiratory signal has 192 channels, and each channel includes 1 × 7 features. The features of each respiratory signal are concatenated to obtain 576 channel features, which are the input of the multichannel attention fusion block. We recalibrate the multichannel features as follows.

First, the *F*_sq_ ( ) operation compresses the features along the spatial dimension, turning each two-dimensional feature channel into an actual number. The global average pooling completes this operation to make the actual number have a global receptive field. The output dimension is the same as the number of input channels. *F*_sq_ (*μ*_*c*_) is calculated as follows:

(1) $$\begin{array}{c} z_{c}=F_{sq}\left(\mu_{c}\right)=\frac{1}{H\times W}\overset{H}{\underset{i=1}{\sum }}\overset{W}{\underset{j=1}{\sum }}\mu_{c}\left(i,j\right)\text{,} \end{array}$$

where *μ*_*c*_ represents the feature map of the *c*-th channel feature map and *i* and *j* represent the row and column of the feature map, respectively.

Second, the *F*_ex_ ( ) operation is similar to the gate mechanism in the recurrent neural network (RNN). This operation can learn a nonlinear interaction between channels, and it can learn a nonmutually exclusive relationship. The operation is completed by two fully connected layers (FC). *F*_ex_ (*z, W*) is calculated as follows:

(2) $$\begin{array}{c} s=F_{ex}\left(z,W\right)=\sigma \left(W_{2}\delta \left(W_{1},z\right)\right)\text{,} \end{array}$$

where *δ* refers to the ReLU function and the parameter *W*_*1*_ multiplied by *Z* is the first FC layer. To limit model complexity and aid generalization, dimensions are reduced according to c/16 × *c*. A dimensionality-increasing layer returns to the channel dimension of the transformation output.

(3) $$\begin{array}{c} X_{c}=F_{re}\left(u_{c},s_{c}\right)=u_{c}{\cdot s}_{c}\text{.} \end{array}$$

Finally, the *F*_re_ ( ) operation regards the output weight of the excitation as the importance of each feature channel. Then, the original feature is recalibrated on the channel dimension by weighting the previous feature by channel. *F*_re_ (*μ*_*c*_, *s*_*c*_) is calculated.where *s*_*c*_ indicates the importance of the feature channel, and *μ*_*c*_ represents the feature map of channel *C*.

After recalibration, there are 576 channel feature maps. The size of each feature map is 1 × 7. After two convolutions and one pooling operation, the convolution kernel sizes are (1, 3) and (1, 2), and the strides are 3 and 2, respectively. The max-pooling size is (1, 2), and the stride is 2. Finally, the flatten operation obtains the 576 features. Then, two fully connected layers and the sigmoid function output the probability of each sleep event. According to the probability value, this block outputs the sleep events.

### 2.5. Performance Evaluation

We evaluate and compare the performance of different methods using classification accuracy, sensitivity (recall), specificity, precision, and *F*1 score. They are defined as follows:

(4) $$\begin{array}{c} A\text{cc}uracy=\frac{TP+TN}{TP+TN+FN+FP}\times 100\%\text{,}\\ S\text{pe}cificity=\frac{TN}{TN+FP}\times 100\%\text{,}\\ Precision=\frac{TP}{TP+FP}\times 100\%,\\ Sensitivity\left(Recall\right)=\frac{TP}{TP+FN}\times 100\%,\\ F1=\frac{Precision*Recall}{Precision+Recall}\times 100\%, \end{array}$$

where TP, FP, TN, and FN represent the number of true positive, false positive, true negative, and false negative epochs. The proportion of the correctly identified epochs is measured by sensitivity. Specificity reflects the detection effect of negative samples.

The confusion matrix also is used. Each row of the confusion matrix represents the epoch in actual labels, while each column represents the epoch in the predicted labels. We also standardized the confusion matrix by rows to obtain different probabilities. We use colors with different shades to represent the probability. The darker the color, the greater the probability, vise versa.

## 3. Experimental Results

This section presents the experimental setup and several experimental results designed to demonstrate the role of each block. First, we showed the classification results of the MCFN model, which proves that the model has better performance. Second, we confirmed the effect of different respiratory signals on different sleep event detections. They complement each other in the SAS detection. Third, we demonstrated the advantages of the multilevel feature concatenation block. Finally, we confirmed that the attention mechanism effectively fuses the multichannel features to improve performance.

### 3.1. Experimental Setup

The proposed network was trained and tested on the MESA dataset. After preprocessing, we selected 1801 subjects from 2506 subjects. They included the 54517 OSA events, 209910 hypopnea events, and 2019760 normal sleep events. The training and test set consisted of a balanced number for each sleep event to prevent the model from overfitting to the majority number of the class. We randomly selected 54517 sleep events from each sleep classification and mitigated the class imbalance issue. The experiment chose 80% of the sleep events as the training set and 20% as the testing set.

The training and testing are conducted based on the TensorFlow framework of Python 3.6. The experiments used the graphics card NVIDIA GTX 2080Ti GPU. The proposed network adopted the Adam optimization method and cross-entropy as the loss function. The initial learning rate is 1*e* − 3, and the learning rate is 1*e* − 4 after 40 iterations. The size of the mini-batch is 400 sleep events. The network had training of 100 epochs.

### 3.2. SAS Detection Performance of MCFN

The MCFN model detects sleep events using three respiratory signals of the chest, abdomen, and nasal airflow on the MESA dataset. The average accuracy is 87.3%, and the average *F*1 score is 87.3%.  Table 2 presents the detection performance of the model. We found that the performance indexes of OSA sleep event detection are the highest, recall can reach 93.7%, the *F*1 score is 93.5%, and precision is 93.3%, indicating that the MCFN model can achieve good performance in detecting OSA events. There is a contradiction between the precision and recall of normal sleep and hypopnea events, which the *F*1 score can measure. The *F*1 scores of the two events are very similar, with a difference of only 0.8%, indicating that the performance of the MCFN model in detecting these two events is the same. From the confusion matrix, we found that there are some misclassifications between normal sleep and hypopnea events, mainly because sometimes the waveforms of the two events are very similar, but there are differences in amplitude. The MCFN model can achieve good performance in detecting OSA events. The main reason is that the waveform of the respiratory signal of OSA events is very different from that of other events.

### 3.3. The Effects of Three Respiratory Signals

We used sensitivity and specificity to measure the effect of different respiratory signals on various sleep events. The sensitivity measures the proportion of correctly identified positives, such as the percentage of OSA events correctly identified as having the event. The specificity measures the proportion of correctly identified negatives, such as the percentage of not OSA correctly identified as not having the event.

We show the sensitivity of airflow (Flow), thoracic respiratory signal (Thor.), and abdominal respiratory signal (Abdo.) in Figure 3. The sensitivity of abdominal respiration signal in detecting OSA and hypopnea sleep events is 81.39% and 73.05%, respectively. The sensitivity of the airflow respiration signals in detecting normal sleep events is 72.9%, which was higher than the other respiratory signals.

We show the specificity in Figure 4. The specificity of the airflow respiratory signal in detecting OSA was 93.72%, and the specificity of detecting hypopnea sleep events was 87.64%, which was 4.31% higher than that of the abdominal respiratory signal. The specificity of abdominal respiratory signals in detecting normal sleep events was 47.2%. These experimental results show that different respiratory signals play different roles in detecting various sleep events, so we can use three respiratory signals simultaneously for SAS detection.

To comprehensively evaluate the role of three respiratory signals in detecting SAS, we show the accuracy in Figure 5. We input single, two, and three respiratory signals into the MCFN model, respectively. It can find that the SAS detection performance of single respiratory signals is the lowest. The accuracy of nasal airflow, abdominal, and thoracic respiratory signals was 76.5%, 76.3%, and 74.0%, respectively. When we combine the respiratory signals in pairs, the accuracy improves to varying degrees compared with that of single respiratory signals, such as the accuracy of combined flow and thoracic respiratory signals which can reach 83.1%, which is 6.6% higher than that of flow. The detection accuracy is the highest when the three respiratory signals are combined, reaching 87.3%. The detection accuracy improved by 9.1%.

We find that the detection performance of the combined respiratory signals is better than that of single respiratory signals. The three kinds of respiratory signals play different roles in detecting sleep events. The combination of multiple respiratory signals can complement each other and improve the SAS detection performance.

### 3.4. Multilevel Features Concatenation Block Improves Performance

In this experiment, we investigate the influence of the multilevel feature concatenation block on classification performances. First, to concatenate the features of different levels, it is necessary to down-sample the shallow features to get the same dimension. There are two methods for down-sampling: average pooling and max pooling. Through the experiment, we find that the two methods have little effect on the detection performance. We choose one way randomly, and here we choose average pooling to reduce the dimension. Then, by inputting different respiratory signals into the model with only deep-level features or multilevel features, the overall accuracy obtained is shown in Figure 6.

We find that whether it is single respiratory signals or combined respiratory signals, the detection accuracy using multilevel features is higher than that using only deep features. For airflow respiratory signals, the accuracy is only improved by 0.2%, indicating that the other level's features provide less identification information. For thoracic respiratory signals, the accuracy with only deep features was 71.1%, and the accuracy with multilevel features was 74.0%. It increased by 2.9%, indicating low-level features of thoracic respiratory signals which can provide rich identification information and improve the detection performance. For the combined respiratory signals, the accuracy can get improvement.

This result shows that the multilevel features of various respiratory signals have different effects on SAS detection. The complete learning features of thoracic and abdominal respiratory signals can improve detection accuracy. In contrast, the multilevel features of airflow respiratory signals have little impact on performance.

### 3.5. Multichannel Features Fusion Block Improves Performance

In this experiment, we investigated the influence of the relationship between different channel features on classification performances. We take two types of airflow and abdominal signals or three kinds of respiratory signals as an example. Whether or not multichannel feature fusion is used, Figure 7 shows the SAS detection confusion matrix.

Comparing the confusion matrices (a) and (b), we find that the correct classification probability of hypopnea events increased from 0.78 to 0.83, increased by 0.05. The correct classification probability of OSA events rose from 0.92 to 0.94, increasing by 0.02. The experimental results show that the respiratory signal combined with abdominal and airflow can extract rich features. After attention fusion, it can strengthen useful features and suppress useless features to improve performance. The correct classification probability of normal sleep events did not increase. Still, it decreased by 0.02, indicating that the extracted features by the two combined signals are very similar.

Comparing the confusion matrices (a) and (c), we find that the correct probability of each event classification in (c) is greater than or equal to that in (a). The experimental results confirm that the classification performance of three respiratory signals is better than that of two signals, which further verifies that various respiratory signals can provide richer information.

Comparing the confusion matrices (c) and (d), we find that the correct probability of event classification in (d) is greater than that in (c). The correct classification probability of hypopnea events increased from 0.82 to 0.86, an increase of 0.04. The correct probability of OSA event and normal event classification has increased by 0.01. The experimental results confirm that the attention mechanism improves the detection performance by fusing the multichannel features of the three respiratory signals.

The abovementioned experimental results confirm that the multichannel attention fusion block can improve the correct classification probability of hypopnea events and OSA events. The effect on normal sleep events is not very significant, mainly because the waveform of such events is relatively stable.

### 3.6. Learned Weight for Each Channel Feature

The attention mechanism can learn different weights for the channel features. The experiment results verify that the channel features of each respiratory signal have different effects on SAS detection.  Figure 8 shows the multichannel feature weights of three respiratory signals. For the first channel of each respiratory signal, the channel weight of airflow respiratory is 0.18, the channel weight of thoracic respiratory is 0.50, and the channel weight of abdominal respiratory is 0.16. For the 64th channel of each respiratory signal, the channel weight of airflow respiratory is 0.50, the channel weight of thoracic respiratory is 0.50, and the channel weight of abdominal respiratory is 0.99. After multilevel feature concatenation of each respiratory signal, the model can obtain 192 channel features. The multichannel feature fusion block obtains 576 channel features. The attention mechanism learns the weight of each feature channel through training.

From Figure 8, we can find that the weights of each respiratory signal feature channel are different. For example, the weights of flow respiratory signals channel features are close to 1, and some are close to 0. These weights indicate that varying levels of features have different effects on sleep event detection. In addition, the weights of the feature channels 0, 32, 64, 96, 128, and 160 are marked with special graphics. The importance of channel features at the same level is also different.

Figure 9 shows the weight distribution of different respiratory signal channel features. When the weight is less than 0.25, the weight distribution of the three respiratory signals is very similar, indicating that the number of weak action feature channels is approximately equal. When the weight is in the range of 0.25∼0.75, the number of feature diagrams of airflow respiratory signal is significant, indicating that the role of airflow respiratory signal is moderately important. When the weight is more powerful than 0.75, the number of the abdominal respiratory signals feature diagrams is large. This result indicates that these features contribute the most to SAS detection and contain the most identifying information. In addition, the Kolmogorov–Smirnov (KS) test further determines whether the channel weights of the two respiratory signals obey the same distribution. Since the *P* values are less than 0.05, they belong to different distributions. Therefore, each respiratory signal learning channel feature has different effects on SAS detection, which shows that the fusion of multiple respiratory signals is essential.

## 4. Discussion

Several methods have been applied to automated sleep event detection in previous studies. They can detect various sleep events, such as OSA, hypopnea, normal sleep, central sleep apnea (CSA), and mixed sleep apnea (MSA). The detection accuracy is compared with previous studies to evaluate the efficiency of MCFN.

Gutiérrez et al. [15] used a single airflow respiratory signal and the AdaBoost method to obtain 86.5% accuracy. They extracted features manually, detected normal sleep and sleep apnea events, and did not classify them in detail. Lin et al. [13] explored the possibility of identifying sleep apnea events, including OSA and CSA, by solely analyzing one or both the thoracic and abdominal respiratory signals. They introduced an adaptive nonharmonic model to model the thoracic and abdominal movement signals. Then, an SVM method was applied to classify three categories of sleep events. When features from the thoracic and abdominal signals were combined, the overall classification accuracy became 81.8%. Jiménez et al. [16] evaluated the complementarity of airflow and oximetry (SpO_2_) signals. They assessed the utility of a multiclass AdaBoost classifier to predict OSA severity in children.

Van Steenkiste et al. [26] used LSTM to detect normal sleep and sleep apnea on large data sets, and the accuracy was 77.2%. Although the temporal correlation of sleep events was considered, they ignored the relationship between different channel features. Elmoaqet et al. [27] developed the LSTM and Bi-LSTM framework to detect apnea events. They evaluated the framework over three respiration signals: airflow, nasal pressure (NPRE), and abdominal respiratory inductance plethysmography. They used PSG recording of 17 patients with obstructive, central, and mixed apnea events. The average accuracy was 83.6%.

Barroso et al. [31] conducted the 13 bispectral features from airflow. The oxygen desaturation index ≥3% (ODI3) was also obtained to evaluate its complementarity to the bispectral analysis. They used the fast correlation-based filter (FCBF) and a multilayer perceptron (MLP) to select the feature and recognize the pattern. The model reached 82.5% accuracy for the typical cut-offs of five events per hour. Yu et al. [32] proposed the SAS detection and classification method, which uses C4/A1 single-channel EEG signal, oronasal flow signal, and abdominal displacement signal. They utilized LSTM-CNN to identify four distinct types: normal sleep, hypopnea events, OSA, and CSA + MSA. The overall classification accuracy achieves 83.94%.

It is challenging to compare as they do not all use the same database and the number of the same sleep classification. To make a comparison on the same dataset, we have implemented the research of Haidar et al., who have carried out a lot of analysis on the MESA dataset. In the beginning, in [22], they got 77.6% accuracy with CNN by inputting airflow respiratory signal. Later, in [23], they obtained 83.5% accuracy by inputting three types of respiratory signals. All the previously mentioned research studies are summarized in Table 3. Considering the effect of shallow features on sleep classification and the relationship between different channel features in detecting sleep events, our experiment improved the accuracy by 3.9%. Our network could not only detect many types of sleep events but also improve accuracy.

## 5. Conclusion

We propose an MCFN model to detect OSA, hypopnea, and normal sleep. The model uses the multilevel feature concatenation block which can extract more rich information and give full play to the role of shallow features. Then, the model utilizes an attention mechanism to effectively fuse the different level features of airflow, abdominal, and thoracic respiratory signals. The fusion block makes each channel feature of three respiratory signals have different weights, enhances the useful channel feature, and suppresses the useless channel feature. The experiments verified that multiple respiratory signals, multilevel features, multichannel fusion, and channel features affect SAS detection. MCFN model improves SAS detection performance by using the complementarity of various signals and the completeness of features. The detection accuracy is 87.3% on the MESA dataset, which is better than the other methods. In future research, we will try to study the effect of sleep apnea on sleep staging.

## Figures and Tables

**Figure 1:** Overall framework of MCFN for SAS detection.

**Figure 2:** Feature maps of different convolution layers. (a) Airflow respiratory signal of OSA. (b) Feature map of the first convolution layer. (c) Feature map of the second convolution layer. (d) Feature map of the third convolution layer. (e) Feature map of the fourth convolution layer.

**Figure 3:** Sensitivity of different respiratory signals on sleep events.

**Figure 4:** Specificity of different respiratory signals on sleep events.

**Figure 5:** SAS detection accuracy of multiple respiratory signal combinations.

**Figure 6:** Influence of multilevel feature block on classification performance.

**Figure 7:** Influence of multichannel feature fusion (MCFF) block on multiple respiratory signals. (a) Two types of respiratory signals without MCFF. (b) Two types of respiratory signals with MCFF. (c) Three types of respiratory signals without MCFF. (d) Three types of respiratory signals with MCFF.

**Figure 8:** Weights of multichannel features of different respiratory signals. (a) Weight of multichannel features on airflow respiratory signal. (b) Weight of multichannel features on the thoracic respiratory signal. (c) Weight of multichannel features on the abdominal respiratory signal.

**Figure 9:** Distribution of weight values on different respiratory signal channel features.

**Table 1:** Parameters in multilevel feature fusion block.

Layer	Size	Stride	#Filter	Activation	Dropout
Conv1	(1, 3)	3	32	ReLU ( )	0.2
Conv2	(1, 2)	2	32	ReLU ( )	0.2
Pooling	(1, 2)	2	32	—	—
Conv3	(1, 3)	3	32	ReLU ( )	0.2
Conv4	(1,2)	2	32	ReLU ( )	0.2
Pooling	(1, 2)	2	32	—	—
Concat	—	—	192	—	—

**Table 2:** Confusion matrix and the per-class result of the MCFN model.

MCFN output							Per-class result (%)
		Normal	Hypopnea	OSA	Precision	Recall	*F*1 score
Ground truth	Normal	4586	836	185	87.5	81.8	84.6
	Hypopnea	574	4842	191	81.4	86.4	83.8
	OSA	79	273	5255	**93.3**	**93.7**	**93.5**

Bold values indicate the highest value of each performance index.

**Table 3:** Performance comparison between MCFN and existing methods.

	Signals	Methods	Patients	Classify	Accuracy (%)
Gutiérrez et al. [15]	Flow	AdaBoost	317	Apnea/normal	86.5
Lin et al. [13]	Flow, Abdo. Thor.	SVM	34	OSA/CSA/hypopnea	81.8
Jiménez et al. [16]	Flow, SpO_2_	AdaBoost	974	OSA/normal	81.3
Haidar et al. [23]	Flow, Abdo. Thor.	CNN	2056	OSA/hypopnea/normal	83.4
Van Steenkiste et al. [26]	Abdo. Thor. EDR	LSTM	2100	Apnea/normal	77.2
Elmoaqet et al. [27]	Flow, Abdo. NPRE	LSTM/Bi-LSTM	17	OSA/CSA/MSA	83.6
Barroso et al. [31]	Flow, ODI3	MLP	946	Apnea/normal	82.5
Yu et al. [32]	EEG, flow, Abdo.	LSTM_CNN	126	Normal/hypopnea/OSA/MSA	83.9
Ours	Flow, Abdo. Thor.	MCFN	2056	OSA/Hypopnea/normal	87.3

## Data Availability

The MESA sleep dataset was supported by the National Heart, Lung, and Blood Institute (NHLBI) at the National Institutes of Health. It is available through NHLBI National Sleep Research Resource at https://www.sleepdata.org/datasets/mesa.
